# Meta-Analysis of the Efficacy and Safety of Olanzapine versus Clozapine when Treating Senile Dementia

**DOI:** 10.1155/2022/5046761

**Published:** 2022-08-11

**Authors:** Zongqin Wang, Yingying Feng, Yanyan Wang, Hui Qiu, Zhongyang Rui, Mingxing Li, Lihua Lv

**Affiliations:** Wuhan Mental Health Center, No. 93 Youyi Road Qiaokou District, China

## Abstract

**Objective:**

To systematically assess the safety and efficacy of olanzapine versus clozapine when treating senile dementia and to provide evidence-based medicine basis for its promotion and use.

**Methods:**

PubMed, Embase, ScienceDirect, Cochrane Library, China Knowledge Network Database (CNKI), China VIP Database, Wanfang Database, and China Biomedical Literature Database (CBM) online database were searched for randomized controlled trials (RCT) of olanzapine and clozapine when treating senile dementia. The retrieval time limit is from the establishment of the database to the present. The data were extracted independently by two researchers, and the bias risk of each contained literature was analyzed in accordance with the standard of Cochrane Handbook 5.3. RevMan 5.4 statistical software was used to analyze the collected data by meta-analysis.

**Results:**

Finally, 6 randomized controlled trial articles were included, with a total of 490 samples. Meta-analysis of clinical efficacy showed that the clinical efficacy was similar and there was no significant difference (*P* > 0.05). Two articles used Alzheimer's disease pathological behavior rating scale (BEHAVE-AD) to compare the pathological behavior of different stages after treatment. Statistical analysis showed that there was no significant difference between the total score of BEHAVE-AD and the scores of each factor in each week after treatment. The non-treatment adverse reaction scale (TESS) of the study group and the control group was analyzed by meta-analysis. The TESS score of the study group after treatment was significantly lower than that of the control group. The BPRS scores of different stages after treatment were analyzed by meta-analysis, and there was no significant difference in the total score and factor scores of BPRS in each week after treatment. Two clinical trials reported the incidence of neurological symptoms after treatment. Olanzapine and clozapine treatment can effectively reduce the risk of aging. There was no significant difference in the incidence of neurological symptoms in patients with dementia (*P* > 0.05). According to the analysis of meat products, the incidence of adverse reactions in the study group was significantly lower than that in the control group (*P* < 0.05).

**Conclusion:**

Olanzapine and clozapine have similar efficacy when treating mental and behavioral disorders in patients with senile dementia, in which olanzapine is more effective in improving the symptoms of patients with Alzheimer's disease (AD), with less adverse reactions and high safety, which is worth popularizing in clinical practice. However, more studies and follow-up with higher methodological quality and longer intervention time are needed to further verify.

## 1. Introduction

There is a progressive and fatal neurodegenerative disease known as Alzheimer's disease (AD), with symptoms of continuing cognitive and memory deterioration, progressive impairment of daily living abilities, and various neuropsychiatric and behavioral dysfunctions [1]. Its pathogenesis is mainly caused by choline deficiency, resulting in memory loss, loss of orientation, behavior and personality changes, and so on. The disease is a common chronic encephalopathy syndrome in the elderly, showing a chronic or progressive process. Because senile dementia patients are accompanied by depression, aggression, hallucinations, and delusions and other so-called mental and behavioral symptoms (BPSD), the use of antipsychotics is inevitable [2]. More than 75% of people with dementia require the care of family members or friends [3, 4]. Dementia with Lewy bodies, AD, cerebral vascular dementia, frontotemporal dementia, and Parkinson's disease dementia are among the most common types of dementia.

Mental and behavioral symptoms of dementia behavioral and psychological symptoms of dementias (BPSD) were defined in 1996 as disorders of perception, emotion, thought content, or behavior [5]. BPSD is a major symptom of dementia, and almost all patients with dementia have at least one BPSD symptom in the course of the disease. The common symptoms of BPSD include depression, hallucination, delusion, anxiety, apathy, irritability, agitation, disinhibition, and sleep behavior disorder. Patients can have a variety of symptoms at the same time or only one. The symptoms that appear in different periods of dementia may be different, and the symptoms of different types of dementia also have their own emphasis. Some studies have confirmed that more than 90% of AD patients develop at least one BPSD symptom at some point in the course of the disease [6, 7]. The commonly used scales for evaluating BPSD are BEHAVE-AD, NPI, Cohen-Mansfield agitation questionnaire, noncognitive part of Alzheimer's disease rating scale (ADAS), and so on. The appearance of BPSD is one of the main reasons for patients with dementia to seek medical treatment, which often means the progression of the disease, resulting in higher mortality. BPSD seriously affects the life quality of patients and their families and brings greater life pressure to patients and caregivers. They contribute to the ill health of countless patients, and these symptoms are the most complex and expensive aspects of care. Studies have shown that one-third of dementia care costs are due to the management of these symptoms, such as the need for additional medical resources, the cost of care, and the cost of additional care [8, 9]. The emergence of BPSD not only noticeably increases the cost of care and treatment but also has a close relationship with the decline in the quality of life, income, stress, and depression of caregivers. Caregivers managing patients with psychobehavioral symptoms of dementia are more distressed or frustrated than caregivers managing patients with dementia alone or with other chronic medical conditions [10].

Common causes of BPSD include unmet patient needs, caregiver factors, environmental triggers, and their interactions. Mechanistic considerations are related to disruption of brain networks, alterations in neurotransmitters. Common methods of treatment of BPSD are nondrug and drug therapy. Nondrug treatments include self-maintenance therapy, memory therapy, music therapy, aromatherapy, physical therapy, light therapy, touch therapy, and integrative therapy. The types of drug treatment include antipsychotic drugs, anticholinesterase drugs, excitatory amino acid receptor antagonists, antidepressants, antiepileptic drugs, and benzodiazepines. Among them, antipsychotics are the most widely used clinically. Typical antipsychotic drugs are chlorpromazine, haloperidol, and so on. The common atypical antipsychotic drugs are risperidone, olanzapine, quetiapine, clozapine, aripiprazole, aminosulfonyl, sulpiride, and so on. The common adverse reactions of antipsychotics are drowsiness, fatigue, dizziness, extrapyramidal symptoms, irritation, psychiatric symptoms, deterioration of cognitive performance, thromboembolism, aspiration pneumonia, metabolic abnormalities, falls, death, and so on. The adverse reactions of typical antipsychotics are more obvious than those of atypical antipsychotics, so atypical antipsychotics are more commonly used.

At present, the efficacy and safety of antipsychotics when treating mental and behavioral symptoms of dementia are still being explored. A systematic analysis showed that there exhibited no remarkable difference in the efficacy of olanzapine, risperidone, and quetiapine when treating BPSD, while quetiapine had the lowest incidence of extrapyramidal symptoms and the lowest incidence of somnolence adverse reactions of risperidone [11]. Recent studies support risperidone and olanzapine as the first choice to treat psychotic and invasive symptoms in patients with dementia [12]. Olanzapine and risperidone are the main atypical antipsychotic drugs. Randomized trials comparing olanzapine and risperidone directly show that olanzapine is more effective than risperidone, and its safety is higher [13]. However, there exhibits no remarkable difference in the therapeutic effect between olanzapine and risperidone, but olanzapine takes effect faster and the incidence of extrapyramidal symptoms is lower [14]. Therefore, this study makes a systematic, quantitative, and comprehensive analysis of the results of similar independent studies through meta-analysis, in order to assess the safety and efficacy of olanzapine versus clozapine when treating senile dementia and provide objective basis for clinical application.

## 2. Research Contents and Methods

### 2.1. The Sources and Retrieval Methods of Documents

We searched PubMed, Embase, ScienceDirect, Cochrane Library, China Journal full-text Database (CNKI), VIP full-text Database (VIP), Wanfang Database, and Chinese Biomedical Literature Data (CBM); searched relevant Chinese journals, conference papers, degree papers, etc.; and collected relevant data about olanzapine and clozapine when treating senile dementia in China. Literature retrieval was conducted in the form of free words and subject words with the keywords of olanzapine, clozapine, AD, effectiveness, safety, meta-analysis, etc., from January 2010 to May 2022.

### 2.2. Literature Inclusion Criteria and Exclusion Criteria

#### 2.2.1. Literature Inclusion Criteria

The inclusion criteria were as follows: (1) type of study: all randomized controlled trials (RCT) of olanzapine and clozapine when treating senile dementia in China; the language is limited to Chinese; (2) subjects: all the patients met the diagnostic criteria of AD, and the score of the pathological behavior rating scale of AD was more than 8 points. There were no antipsychotic drugs and no somatic diseases before this trial. No other antipsychotic drugs were used during treatment; (3) intervention: the study group was cured with olanzapine, and the control group was cured with clozapine.

#### 2.2.2. Literature Exclusion Standard

The exclusion criteria were as follows: (1) it is not a randomized controlled study; (2) the data report is incomplete, and the data cannot be used; (3) repeat the research content, and take the latest research; (4) the evaluation of the curative effect of the study was not remarkable.

### 2.3. Quality Evaluation and Data Extraction

1. Bias risk assessment contained in the study: the bias risk assessment tool recommended by Cochrane System Review Manual 5.3 was used for evaluation
2. Identifying the literature and collecting data: two researchers independently identify the literature, collect the data, evaluate the quality, and cross-check. Whenever there are differences, discuss them and resolve them, or ask the third researcher for assistance. Of note, Express document management software and Excel Office software were used to manage and extract research data. If the data contained in the literature is incomplete, contact the author of this article to supplement it. The content of data extraction contains (1) basic information: writer, number of cases, and publication time; (2) intervention: plan and course of treatment; and (3) outcome index

### 2.4. Statistical Processing

The RevMan 5 software originated from Cochrane collaboration network for meta-analysis. The mean and standard deviation of the net change difference of serum albumin, prealbumin, and hemoglobin in the experiment and the control cohorts were input into RevMan 5 for analysis. Because the index is a continuous variable, the weighted mean difference (WMD) is used as the effect scale, and 95% confidence interval is selected. First, the *X*^2^ test is used to determine whether there is heterogeneity between the studies; if *P* > 0.05 and *I*^2^ < 50%, it is considered that the included study is homogeneous, and the modified impact model can be collected for meta-analysis. If *P* < 0.05 and *I*^2^ ≥ 50%, when judging the homogeneity of the included study, the combined effect is needed, then choose the random effect model. If *P* < 0.05 and the source of heterogeneity could not be judged, meta-analysis was not performed, and descriptive analysis was used.

## 3. Results and Analysis

### 3.1. The Results of Literature Retrieval and the Basic Situation of Literature Inclusion

1321 articles were retrieved through computer database; 526 articles were obtained after eliminating repeated studies; 271 articles were obtained by preliminary reading of titles and abstracts; 93 articles were contained after excluding irrelevant studies, reviews, case reports and noncontrol literatures; and then, 87 articles with incomplete data and no main outcome indicators were read carefully and finally contained 6 RCTs [15–20]. A total of 490 samples were analyzed by meta-analysis. The basic features contained in the literature are shown in Table 1.

### 3.2. Evaluation of the Quality of the Methodology Contained in the Literature

The 6 RCTs contained in this meta-analysis are all reported on the patients' baseline conditions. One of the RCTs did not mention “random assignment.” The six contained studies gave detailed intervention measures and treatment duration. None of the 6 RCTs described in detail the number and reasons for blinding and loss to follow-up or withdrawal. According to the Jadad scale, it can be seen that the 6 RCTs are all ≤2 points. The risk bias analysis is shown in Figures 1 and 2.

### 3.3. Meta-Analysis Result

#### 3.3.1. Clinical Curative Effect

A total of 6 RCT studies were contained in this study, with a total of 490 samples, and a meta-analysis was conducted on the clinical efficacy. The results of the heterogeneity test showed that chi^2^ = 0.50, df = 3, *P* = 0.92, and *I*^2^ = 0%, indicating that there is no obvious heterogeneity among the contained research data. According to the analysis in Figure 3, the clinical efficacy is comparable, and the difference was not statistically significant (*P* > 0.05), suggesting that olanzapine and clozapine have similar efficacy for the treatment of mental and behavioral disorders in patients with AD.

#### 3.3.2. Alzheimer's Disease Pathological Behavior Score Scale (BEHAVE-AD)

A total of 6 RCT studies were contained in this study, with a total of 490 samples, of which 2 articles used the AD pathological behavior rating scale (BEHAVE-AD) to compare the pathological behavior at different stages after treatment, from the heterogeneity test results: 2 weeks after treatment: chi^2^ = 4.90, df = 15, *P* = 0.99, and *I*^2^ = 0%; four weeks after treatment: chi^2^ = 1.02, df = 15, *P* = 1.00, and *I*^2^ = 0%; eight weeks after treatment: chi^2^ = 1.10, df = 15, *P* = 1.00, and *I*^2^ = 0%. It shows that there is no obvious heterogeneity among the contained research data. From the analysis of Figures 4–6, it can be noticed that there exhibits no remarkable difference in the total score of BEHAVE-AD and each factor score after each week of treatment (*P* > 0.05), suggesting that olanzapine and clozapine have similar effects on the improvement of pathological behavior in patients with senile dementia.

#### 3.3.3. Adverse Drug Reaction Scale (TESS)

A total of 6 RCT studies were contained in this study, with a total of 490 samples. A meta-analysis was carried out on the treatment-free adverse reaction scale (TESS). The results of the heterogeneity test showed that after 2 weeks of treatment, chi^2^ = 0.00, df = 1, *P* = 0.96, and *I*^2^ = 0%; after 4 weeks of treatment, chi^2^ = 1.00, df = 1, *P* = 0.32, and *I*^2^ = 0%; and after 8 weeks of treatment, chi^2^ = 0.75, df = 2, *P* = 0.69, and *I*^2^ = 0%. A summary analysis of all the literatures was carried out, and the results of the heterogeneity test showed the following: chi^2^ = 6.22, df = 6, *P* = 0.40, and *I*^2^ = 3%, indicating that there exhibits no obvious heterogeneity among the contained research data, and the analysis in Figure 7 shows that the TESS score of the study group was noticeably lower compared to that of the control group after treatment, and the difference was statistically significant (*P* < 0.05), suggesting that compared with clozapine, the incidence of adverse reactions of olanzapine when treating senile dementia patients was lower.

#### 3.3.4. Concise Psychiatric Rating Scale (BPRS)

A total of 490 RCT studies were contained in this study, and the BPRS scores at different stages after treatment were meta-analyzed. According to the heterogeneity test results, after 2 weeks of treatment, chi^2^ = 0.14, df = 1, *P* = 0.71, and *I*^2^ = 0%; after 4 weeks of treatment, chi^2^ = 1.49, df = 1, *P* = 0.22, and *I*^2^ = 33%; and after 8 weeks of treatment, chi^2^ = 1.66, df = 1, *P* = 0.20, and *I*^2^ = 40%. A summary analysis of all the literatures was carried out, and the results of the heterogeneity test showed the following: chi^2^ = 4.19, df = 5, *P* = 0.52, and *I*^2^ = 0%, indicating that there exhibits no obvious heterogeneity among the contained research data, and the analysis in Figure 8 shows that there exhibited no remarkable difference in the BPRS total score and each factor score in each week of treatment (*P* > 0.05), which indicates that olanzapine can help reduce the mental symptoms of patients and promote patients.

#### 3.3.5. Incidence of Neurological Symptoms

A total of 6 RCT studies were contained in this study, with a total of 490 samples, of which 2 clinical trials reported the incidence of neurological symptoms after treatment. The results of the heterogeneity test showed the following: delusions/hallucinations: chi^2^ = 0.32, df = 1, *P* = 0.57, and *I*^2^ = 0%; abnormal behavior: chi^2^ = 1.30, df = 1, *P* = 0.25, and *I*^2^ = 23%; and anxiety and depression: chi^2^ = 1.72, df = 1, *P* = 0.19, and *I*^2^ = 0%, indicating that there exhibits no obvious heterogeneity among the contained research data; from the analysis in Figure 9, it can be noticed that both olanzapine and clozapine treatments can successfully reduce the incidence of neurological symptoms in senile dementia patients, and the difference was statistically significant (*P* > 0.05), which suggests that olanzapine and clozapine are effective in elderly patients. The improvement of neurological symptoms in patients with stage dementia was comparable.

#### 3.3.6. Adverse Reaction

A total of 6 RCT studies were contained in this study, with a total of 490 samples. Meta-analysis was conducted on the occurrence of adverse reactions of patients after treatment. Common adverse reactions include drowsiness, salivation, weight gain, dizziness, and rapid heart rate. A summary analysis of all the literatures was carried out, and the results of the heterogeneity test showed the following: chi^2^ = 10.26, df = 19, *P* = 0.95, and *I*^2^ = 0%, indicating that there exhibits no obvious heterogeneity among the contained research data. The analysis in Figure 10 shows that the incidence of adverse reactions in the study group after treatment was noticeably lower compared to that in the control group, and the difference was statistically significant (*P* < 0.05), suggesting that compared with clozapine, the incidence of adverse reactions in patients with senile dementia treated with olanzapine was lower.

## 4. Analysis and Discussion

Senile dementia is the general name of all kinds of senile dementia, mainly including AD and vascular dementia (VD). Its clinical manifestations are the continuous deterioration of cognitive and memory function, the progressive decline of the ability of daily life, and various behavioral disorders and neuropsychiatric symptoms. In clinical, it is characterized by intellectual impairment. In addition, Alzheimer's is also the fourth leading cause of disability and death in the elderly after tumors and cardiovascular and cerebrovascular diseases. Approximately 44 million people lived with dementia worldwide in 2013, according to statistics. There will be 76 million people with dementia in 2030 and 135 million in 2050, according to estimates [21]. Because the senile dementia patient is older, the liver and kidney functions are decreased; the drug absorption is slow; the excretion is prolonged; because of the increased sensitivity to the drug, it is easy to produce all kinds of adverse reactions; and most senile dementia patients are accompanied by somatic diseases, especially cardiovascular diseases, so the treatment of senile dementia patients with mental symptoms should not only consider the efficacy but also consider the safety of drugs [22].

There are many clinical methods to treat BPSD. The commonly used drugs for the treatment of mental and behavioral symptoms are anticholinesterase drugs, excitatory amino acid receptor antagonists, antipsychotic drugs, antidepressant drugs, antiepileptic drugs, benzodiazepine drugs, and so on. The most commonly used and effective atypical drugs are olanzapine, risperidone, and quinosulfan equality. Studies have shown that olanzapine, clozapine, and risperidone are superior to placebo when treating mental and behavioral symptoms of dementia, and quetiapine does not show a remarkable advantage over placebo [23, 24]. The aim of this study was to compare the safety and efficacy of olanzapine and clozapine when treating mental and behavioral symptoms of dementia. Through a comprehensive search of some databases, collection of relevant literature, formulation of inclusion and exclusion criteria, screening of literature, and quality evaluation of the article, a total of 6 articles with sample size of 490 cases were contained, and the relevant data were extracted. Finally, statistical analysis was carried out by RevMan 5.3 software.

Olanzapine is an antipsychotic drug with pharmacological effects on a variety of receptor systems, with affinity for 5-HT, dopamine D, *α*-adrenergic, histamine H, and other receptors, as well as dopamine and choline. It can antagonize and even selectively reduce the firing of dopaminergic neurons in the limbic system (A10), while having little effect on the motor function pathway of the striatum (A9) [25–27]. Meta-analysis showed that the clinical efficacy was similar and there was no significant difference between olanzapine and clozapine in the treatment of mental and behavioral disorders in patients with AD. The meta-analysis of the concise psychiatric rating scale at different stages after treatment showed that there was no significant difference in the total score and factor scores of BPRS in each week after treatment, suggesting that olanzapine can help patients with mental symptoms and improve their daily behavior. Two articles were compared with Alzheimer's disease pathological behavior rating scale (BEHAVE-AD). There was no significant difference in the total score and factor scores of BEAHAVE-AD in different weeks after treatment, suggesting that olanzapine and clozapine have similar effects on pathological behavior in patients with senile dementia. Meta-analysis of the incidence of neurological symptoms showed that there was no significant difference between olanzapine and clozapine, suggesting that olanzapine and clozapine can improve the neurological symptoms of senile dementia. The effect is comparable. It shows that olanzapine has obvious advantages over clozapine in these aspects and affirms its role in improving patients' living ability and intelligence. This may be related to the prominent role of olanzapine in serotonin, dopamine, and cholinergic antagonism, so its effect on neurotransmitter improvement is obvious.

However, it is worth noting that olanzapine also has certain side effects, such as drowsiness, weight gain, and dizziness. Its clinical manifestations are mild, but it still needs to be paid enough attention in the process of treatment [28–30]. A meta-analysis was carried out on the treatment-free adverse reaction scale (TESS). The results of the heterogeneity test showed that after 2 weeks of treatment, chi^2^ = 0.00, df = 1, *P* = 0.96, and *I*^2^ = 0%; after 4 weeks of treatment, chi^2^ = 1.00, df = 1, *P* = 0.32, and *I*^2^ = 0%; after 8 weeks of treatment, chi^2^ = 0.75, df = 2, *P* = 0.69, and *I*^2^ = 0%. A summary analysis of all literatures was carried out, and the results of the heterogeneity test showed the following: chi^2^ = 6.22, df = 6, *P* = 0.40, and *I*^2^ = 3%, indicating that there exhibited no obvious heterogeneity among the contained research data. The analysis showed that in the research group after treatment, the TESS score was noticeably lower compared to the control group (*P* < 0.05), showing that compared with clozapine, the incidence of adverse reactions in olanzapine when treating senile dementia was lower. Previous studies have found that small doses can achieve better efficacy, but the incidence of adverse reactions can be effectively reduced, suggesting that attention should be paid to clinical dosage. There are some limitations in this study. First of all, the sample size of the references included in this study is small, and they all belong to single-center research; there is a certain deviation. In the future research, we will carry out a large sample of prospective studies and hopefully draw more valuable conclusions.

## 5. Conclusion

To sum up, olanzapine and clozapine are effective when treating mental and behavioral symptoms of senile dementia, but olanzapine has less side effects and is more suitable for the treatment of senile dementia with mental symptoms than clozapine in terms of safety.

## Figures and Tables

**Figure 1:** Risk of bias.

**Figure 2:** Risk of bias summary.

**Figure 3:** Forest plot of meta-analysis of clinical efficacy.

**Figure 4:** Forest plot of meta-analysis of BEHAVE-AD scale score.

**Figure 5:** Forest plot of meta-analysis of BEHAVE-AD scale score.

**Figure 6:** Forest plot of meta-analysis of BEHAVE-AD scale score.

**Figure 7:** Forest plot of meta-analysis of TESS score.

**Figure 8:** Forest plot of meta-analysis of BPRS score.

**Figure 9:** Forest plot of meta-analysis of incidence of neurological symptoms,

**Figure 10:** Forest plot of meta-analysis of adverse reactions.

**Table 1:** Basic characteristics of literature.

Include the literature	Year of publication	N (C/T)	Intervention method		Outcome index	Course of treatment	Whether it is random or not	Whether it is blind or not
			C	T				
Wan [15]	2011	38/38	Clozapine	Olanzapine	②⑤	8 weeks	Yes	Yes
Yu et al. [16]	2011	38/38	Clozapine	Olanzapine	②③⑤	8 weeks	Yes	No
Gong [17]	2014	70/70	Clozapine	Olanzapine	⑤	8 weeks	Yes	No
Zhu [18]	2015	26/26	Clozapine	Olanzapine	④⑤⑥	8 weeks	No	No
Xu [19]	2012	50/50	Clozapine	Olanzapine	①③	8 weeks	Yes	No
Kong and Yu [20]	2014	23/23	Clozapine	Olanzapine	①③④⑤	8 weeks	No	No

Note: C: control group; T: research group; ① clinical curative effect; ② BEHAVE-AD scoring; ③ TESS scoring; ④ incidence of mental symptoms; ⑤ adverse reaction; ⑥ BPRS scoring.

## Data Availability

The datasets used and analyzed during the current study are available from the corresponding author upon reasonable request.
